# Influence of Information-Based Continuous Care on Disease Control and Treatment Compliance of Elderly Diabetic Patients

**DOI:** 10.1155/2022/4023123

**Published:** 2022-10-15

**Authors:** Jiao liu, Xiaomao Shi, Bin Guo

**Affiliations:** HunanProvincialPeople's Hospital (The First Affiliated Hospital of the Hunan Normal University), Changsha 410000, Hunan, China

## Abstract

**Background:**

The incidence of diabetes is increasing year by year. For elderly diabetic patients, poor blood glucose control and worsening immune function greatly increase the risk of complications, which will seriously affect their quality of life.

**Purpose:**

This paper primarily clarifies the influence of information-based continuous care on disease control and treatment compliance of elderly diabetic patients.

**Methods:**

From December 2018 to December 2021, 106 elderly diabetic patients were selected, and their clinical data were retrospectively studied. Patients were grouped according to the type of care they received: an observation group (OG) comprising 56 cases receiving information-based continuous care and a control group (CG) including 50 cases treated with routine nursing. The two cohorts of patients were compared regarding disease control, treatment compliance, glucose and lipid metabolism (GLM), and self-management.

**Results:**

After analysis, it was found that the disease control and treatment compliance were statistically higher in OG compared with CG. OG also showed significantly reduced fasting blood glucose (FBG), 2-hour postprandial blood glucose (2hPG), total cholesterol (TC), and triglyceride (TG) after nursing that were all lower compared with CG. In terms of self-management, OG outperformed CG in diet, exercise, blood glucose monitoring, and adherence to medical regimens.

**Conclusions:**

Information-based continuous care has beneficial effects on disease control and treatment compliance of elderly diabetic patients and can help control blood sugar and optimize patients' self-management level, with high clinical promotion value.

## 1. Introduction

Diabetes mellitus (DM) is a chronic metabolic disease, with clinical experience indicating that approximately 95% of all diagnosed cases being type 2 diabetes mellitus (T2DM) and 5% being type 1 diabetes mellitus (T1DM) [1, 2]. Different DM types are generally considered to be related to insulin resistance due to the inability to produce insulin and improper use of glucose (T1DM) or the ability to produce hormones but inability to interact with its receptors (T2DM) [3]. Recent years have witnessed the gradual rise of the incidence of DM. However, the early onset of DM is insidious, and a cure is difficult to achieve after onset [4, 5]. It is shown that for elderly DM patients with vascular fragility, poor blood glucose (BG) control, and deteriorating immune function, there is a higher risk of infective complications, which seriously affects the quality of life of patients and their caregivers [6]. Choosing an appropriate care model is critical due to the great difficulty in curing the disease. This study mainly explores the influence of information-based continuous care on disease control and treatment compliance of elderly DM patients, aiming at optimizing the management mode of such patients, which is of great significance to improve patients' clinical symptoms and their self-management level.

Continuous nursing is a care method that aims to consolidate and maintain treatment effects and attempts to improve disease outcomes through long-term management of patients [7]. The gradual maturity and promotion of the Internet of Things technology makes continuous nursing based on information possible [8]. Under this mode, smart phones can be used as media to provide a series of automatic functions for patients through software, and telephone consultants can also be utilized to provide effective continuity of care for elderly DM patients [9]. In the research of Xia [10], on the influence of information-based continuous nursing on colostomy patients, this nursing method shows obvious advantages in enhancing patients' self-efficacy and confidence, contributing to reduced complications and improved life quality. This report is enlightening. The routine nursing currently applied is not effective in controlling the disease in elderly DM patients, which is mainly because DM is difficult to cure and requires long-term blood glucose management, while long-termin-hospital routine nursing often causes a great economic burden to patients. Considering the above-mentioned conditions, this research is expected to provide a new reference for the management of elderly DM patients by comparing the differences in disease control and treatment compliance between information-based continuous care and routine care.

## 2. Data and Methods

### 2.1. General Information

This retrospective study selected 106 elderly DM patients presented between December 2018 and December 2021 to the Hunan Provincial People's Hospital. According to the type of care they received, they were assigned to two cohorts: an observation group (OG) comprising 56 cases receiving information-based continuous care and a control group (CG) including 50 cases treated with routine nursing.

The mean age and average disease course of OG were (69.45 ± 6.48) years and (7.28 ± 3.51) years, respectively, while those of CG were (68.76 ± 5.54) years and (7.08 ± 3.51) years, respectively. The two cohorts of patients were clinically comparable without statistical differences in general data (*P* > 0.05).

The Ethics Committee of Hunan Provincial People's Hospital approved this research without reservations, and all subjects provided informed consent.

### 2.2. Eligibility Criteria

Elderly patients who were in accordance with the diagnosis of DM and willing to receive follow-up and guidance, with normal communication and cognitive ability, and no mental illness or communication disorders were enrolled.

Those with severe heart, lung, kidney dysfunction, other serious chronic diseases, malignant tumors, or incomplete medical records, and those who refused to participate in this clinical trial were excluded.

### 2.3. Nursing Methods

CG was given routine nursing. Guidance on correct medication and dietary, as well as monitoring of patients' BG and timely management of related complications were given according to the patients' condition.

Information-based continuous care was used in OG: (1) a nursing plan was formulated according to each patient's specific condition. (2) DM health education manual and self-monitoring diary were distributed to each patient. (3) The Internet hospital medical service model was adopted. The Internet was used as an auxiliary tool of extended medical care to provide complete medical support for elderly DM patients in consultation, diagnosis and treatment, drug purchase, rehabilitation nursing, and health management. (4) An information platform was established, and new media such as QQ and WeChat were used to strengthen communication with patients and/or their relatives. (5) Home nursing intervention was also provided, mainly including psychological intervention (patiently listening to patients' demands and timely adjusting patients' state of mind), dietary guidance (guiding patients to calculate daily calories and determining appropriate recipes), and life and health care guidance (preventing colds and cleaning the vulva with warm water). (6) Patients were encouraged to do aerobic exercise (walking, jogging, swimming, Tai Chi, etc.) within 1 to 3 hours after meals at least once every two days. (7) Patients were instructed to correctly use the BG meter to self-monitor BG and to take antihypertensive and hypoglycemic drugs reasonably. The indications, contraindications, and possible adverse reactions of drugs were also introduced to patients. For those with poor compliance or memory, medication supervision was strengthened. (8) Importance was also attached to the follow-up. Home visits were performed at least once every two weeks during the first 3 months following discharge. During the fourth to sixth months, a telephone follow-up at least every half a month and a home visit every month were carried out so as to identify potential adverse factors in time.

### 2.4. Disease Control Efficacy Assessment

Marked improvement: it was defined as FBG <7.2 mmol/L, 2hPG <8.3 mmol/L, TC < 1.8 mmol/L, and TG < 5.3 mmol/L.

Improvement: it was defined as FBG <8.3 mmol/L, 2hPG <10.0 mmol/L, TC < 2.5 mmol/L, and TG < 6.5 mmol/L.

Ineffectiveness: if the patient's BG and glycation control indexes did not meet the above standards, it was classified as ineffectiveness.

### 2.5. Outcome Measures

Nursing efficacy. The assessment criteria for disease control are shown above. The total effective rate of disease control was the percentage of the total number of patients with significant improvement and improvement in the total number of cases.

Treatment compliance. Complete compliance: the patient takes the medicine on time and actively as instructed; compliance: the patient does not take the medicine on time but passively; noncompliance: coercive measures have to be taken to make the patient take medicine because the patient hides the drugs and refuses to take medicine.

Glucose and lipid metabolism (GLM). The information platform was utilized to supervise and guide patients to use BG meters to measure BG and to count the levels of FBG, 2hPG, TC, and TG.

Self-management. The self-management ability scale made by our hospital was used to evaluate the self-management ability of patients from four aspects: active diet control, self-monitoring of BG, active exercise, and adherence to medical regimens.

### 2.6. Statistical Processing

This study used the SPSS21.0 software package for statistical analysis and GraphPad Prism 6 for visualization. The number of cases/percentage (*n*/%) and mean ± SEM were used to represent count data (e.g., sex and smoking history) and quantitative data (e.g., age and disease duration), respectively. As for the methods for comparisons, *χ*^2^ test was used for count data, while the independent sample *t*-test and paired *t*-test were used to identify within-group and between-group differences of quantitative data, respectively, with *P* < 0.05 as the significance level for all tests.

## 3. Results

### 3.1. General Information of Elderly DM Patients

As shown in Table 1, the general data (sex, age, disease course, smoking/alcoholism history, exercise habits, marital status, place of residence, etc.) of the two groups were comparable, with no statistical significance (*P* > 0.05).

### 3.2. Disease Control of Elderly Diabetic Patients

As presented in Table 2, the nursing efficacy was evaluated as significant improvement in 27 cases, improvement in 24 cases, and ineffectiveness in 5 cases in OG, while in CG, the number of significant improvement, improvement, and ineffectiveness cases was 19, 20, and 13, respectively. OG had a statistically higher total effective rate of disease control than CG (91.07% vs. 78.00%, *P* < 0.05).

### 3.3. Treatment Compliance of Elderly Diabetic Patients

We evaluated patients' treatment compliance to analyze the influence of the two nursing methods on treatment compliance (Table 3); the data showed that the corresponding cases of complete compliance, partial compliance, and noncompliance in OG were 23, 30, and 3, respectively, while those in CG were 15, 25, and 10, respectively. The data revealed obviously higher treatment compliance in OG compared with CG (94.64% vs. 80.00%, *P* < 0.05).

### 3.4. GLM in Two Groups

We tested GLM indexes to compare and evaluate the impacts of two intervention models on GLM (Figure 1). Statistical significance was absent in GLM indexes between the groups prior to intervention (*P* > 0.05) while these indexes decreased to varying degrees after intervention, with significantly lower FBG, 2hPG, TC, and TG in OG versus CG (*P* < 0.05).

### 3.5. Self-Management Level of Elderly Diabetic Patients

We evaluated the self-management level of patients from the aspects of active diet control, active exercise, self-monitoring of BG, and adherence to prescribed medication (Table 4). It was found that the self-management level of OG was significantly better than that of CG in these four aspects (*P* < 0.05).

## 4. Discussion

Against the background of socioeconomic development and population aging trend, the incidence of DM in the elderly is increasing year by year [11]. It has been reported that elderly DM patients are more predisposed to osteoporosis and chronic cardiopulmonary diseases [12, 13]. According to statistics, the prevalence of osteoporosis in elderly T2DM patients is as high as 31.7%, which seriously hinders the normal life activities of such patients and greatly affects patients' as well as their families' quality of life [14]. Therefore, optimizing nursing methods is of great significance for improving the outcome and quality of life of elderly DM patients.

With the increase in the number of patients, the working pressure on nurses in hospital is also increasing [15]. For elderly DM patients with high risk of recurrence, it is necessary to maintain long-term continuous care after the initial stage of intensive treatment [16]. Among the several new approaches with favorable application that can provide continuity of care for patients, the information-based continuous care model provides patients with longer continuous care while actively engaging them, which may produce more positive outcomes for patients [17]. This study included 106 elderly DM patients as the research subjects and divided into an OG (information-based continuous care) and a CG (routine nursing care) according to the nursing models. In our research, markedly better disease control was observed in OG, indicating that information-based continuous care has a significant impact on the disease control of elderly DM patients. In the report on the application of information-based continuous nursing in patients with coronary heart disease, Zhou et al. [18] indicated that this nursing method can effectively reduce the risk of disease under exposure to various risk factors and avoid disease recurrence and deterioration, which is consistent with the results of disease control in this study. Then, we detected GLM indicators in both groups of patients. The results determined statistically lower GLM indexes FBG, 2hPG, TC, and TG in OG, suggesting that it was more advantageous to adopt information-based continuous care in glucose and lipid control. FBG and 2hPG can directly reflect the BG level of patients, while TC and TG have been proved to be linked to the incidence of DM in previous studies, and the abnormal increase of the two is a risk factor for the onset of DM in elderly patients [19, 20]. The reduction of the above four indicators demonstrates that information-based continuous care exerts a positive impact on the disease control of elderly DM patients. In the nursing plan of the observation group, we guided patients to use the BG meter to detect the BG level through the information platform and supervised patients to take drugs reasonably, so the BG level of patients was well controlled. In addition, we also arranged aerobic exercise at least once every two days. In the report of Mehbodniya et al. [21], it was suggested that aerobic exercise could affect patients' lipid metabolism, which in turn effectively reduced patients' TC and TG levels, similar to our findings. Later, we evaluated patients' performance in terms of treatment compliance. After analysis, it was found that OG had markedly higher treatment compliance than CG (94.64% vs. 80.00%), which suggested that information-based continuous care is helpful to improve the treatment compliance of elderly DM patients. This may be due to the distribution of education manuals and self-test diaries to patients in the observation group to lay the foundation for patients' compliance with treatment; in addition, medical staff maintain communication with patients and their families through the information platform and timely communicate with patients once they are found to have negative emotions, which all lead to the improvement of patients' treatment compliance. By evaluating the self-management level of the two groups of patients, we found that OG outperformed CG in the aspects of diet control, exercise, self-monitoring of BG, and adherence to prescribed medication, demonstrating that information-based continuous care can help optimize patients' self-management level. Mehbodniya et al. [22] pointed out in their study on information-based nursing for DM control and self-management that information-based medical management has a bright future in promoting self-health care and self-management.

The innovation of this research lies in the comprehensive analysis of the intervention effect of information-based continuous nursing from the aspects of disease control, treatment compliance, GLM, and self-management level of patients, which confirms its effectiveness in elderly DM patients and provides a new choice for nursing management of such patients. But there is still a room for improvement in this study. First of all, only 106 samples were included for analysis, so the number of subjects needs to be expanded to improve the accuracy of the conclusions. Second, this study is a single-center study, which is prone to information bias. Finally, due to the limitation of objective conditions, some corresponding indicators of elderly DM patients have not been studied. In the future, we will improve the research from the above perspectives.

Conclusively, information-based continuous care can better control the condition of elderly DM patients and effectively improve their treatment compliance and self-management level, which is conducive to disease management and is worth popularizing in clinics.

## Figures and Tables

**Figure 1:** Glucolipid metabolism in two groups. (a) FBG of patients in both groups. (b) 2hPG of patients in both groups. (c) TC of patients in both groups. (d) TG of patients in both groups. Note: ^*∗*^means *P* < 0.05 compared with the level before treatment (intragroup); ^#^means *P* < 0.05 between the observation group and the research group after treatment *P* < 0.05. FBG, fasting blood glucose; 2hPG, 2 hours postprandial blood glucose; TC, total cholesterol; TG, triglyceride.

**Table 1:** General data of elderly diabetic patients (*n* (%), mean ± SEM).

Elements	Control group (*n* = 50)	Observation group (*n* = 56)	*χ* ^2^/*t*	*P*
Gender (male/female)	28/22	34/22	0.242	0.623
Age (years old)	68.76 ± 5.54	69.45 ± 6.48	0.586	0.559
Course of disease (years)	7.08 ± 3.51	7.28 ± 3.51	0.293	0.770
History of smoking (yes/no)	24/26	23/33	0.514	0.474
History of alcoholism (yes/no)	13/37	15/41	0.008	0.927
Exercise habit (yes/no)	10/40	13/43	0.161	0.689
Marital status (married/single)	34/16	39/17	0.033	0.855
Place of residence (urban/rural)	24/26	21/35	1.192	0.275

**Table 2:** Disease control of elderly diabetic patients (*n* (%)).

Groups	*n*	Marked improvement	Improvement	Ineffectiveness	Total effective rate (%)
Control group	50	19 (38.00)	20 (40.00)	13 (26.00)	39 (78.00)
Observation group	56	27 (48.21)	24 (42.86)	5 (8.93)	51 (91.07)
*χ* ^2^ value	—	—	—	—	5.014
*P* value	—	—	—	—	0.025

**Table 3:** Treatment compliance of elderly diabetic patients (*n* (%)).

Groups	*n*	Complete compliance	Partial compliance	Non-compliance	Total compliance
Control group	50	15 (30.00)	25 (50.00)	10 (20.00)	40 (80.00)
Observation group	56	23 (41.07)	30 (53.57)	3 (5.36)	53 (94.64)
*χ* ^2^ value	—	—	—	—	5.264
*P* value	—	—	—	—	0.022

**Table 4:** Self-management level of elderly diabetic patients (*n* (%)).

Groups	*n*	Active diet control	Active exercise	Self-monitoring of blood glucose	Adherence to prescribed medication
Control group	50	32 (64.00)	25 (50.00)	28 (56.00)	33 (66.00)
Observation group	56	50 (89.29)	52 (92.86)	56 (100.00)	48 (85.71)
*χ* ^2^ value	—	9.642	24.413	31.093	5.696
*P* value	—	0.002	<0.001	<0.001	0.017

## Data Availability

The labeled dataset used to support the findings of this study is available from the corresponding author upon request.
